# Mendelian randomization supports a causative effect of TSH on thyroid carcinoma

**DOI:** 10.1530/ERC-20-0067

**Published:** 2020-07-21

**Authors:** Jonathan M Fussey, Robin N Beaumont, Andrew R Wood, Bijay Vaidya, Joel Smith, Jessica Tyrrell

**Affiliations:** 1 Head and Neck Surgery, Royal Devon and Exeter Hospital, Exeter, UK; 2 Genetics of Complex Traits, Institute of Biomedical and Clinical Science, University of Exeter Medical School, Exeter, UK; 3 Endocrinology, Royal Devon and Exeter Hospital, Exeter, UK

**Keywords:** mendelian randomization, thyroid neoplasms, molecular epidemiology, thyrotropin

## Abstract

Evidence from observational studies suggest a positive association between serum thyroid-stimulating hormone (TSH) levels and differentiated thyroid carcinoma. However, the cause–effect relationship is poorly understood and these studies are susceptible to bias and confounding. This study aimed to investigate the causal role of TSH in both benign thyroid nodules and thyroid cancer in up to 451,025 UK Biobank participants, using a genetic technique, known as Mendelian randomization (MR). Hospital Episode Statistics and Cancer Registry databases were used to identify 462 patients with differentiated thyroid carcinoma and 2031 patients with benign nodular thyroid disease. MR methods using genetic variants associated with serum TSH were used to test causal relationships between TSH and the two disease outcomes. Mendelian randomization provided evidence of a causal link between TSH and both thyroid cancer and benign nodular thyroid disease. Two-sample MR suggested that a 1 s.d. higher genetically instrumented TSH (approximately 0.8 mIU/L) resulted in 4.96-fold higher odds of benign nodular disease (95% CI 2.46–9.99) and 2.00-fold higher odds of thyroid cancer (95% CI 1.09–3.70). Our results thus support a causal role for TSH in both benign nodular thyroid disease and thyroid cancer.

## Introduction

Thyroid cancer is the most common endocrine malignancy, with recent years seeing a significant increase in incidence (Kitahara & Sosa 2016). The majority of patients present with a thyroid nodule; however, nodules are common with a prevalence of up to 34% on ultrasound (Moon *et al.* 2018) and only 5–10% of nodules are malignant (Hegedüs 2004, Perros *et al.* 2014). Following clinical assessment, ultrasonography and cytological analysis of fine-needle aspiration biopsy the true nature of the nodule remains indeterminate in up to 25% of cases and up to one-third of surgically excised nodules are in fact benign (Bongiovanni *et al.* 2012). There is, therefore, a need for better stratification of thyroid nodules according to risk of malignancy, and while recent years have seen the development of genomic tests to aid diagnosis (Nikiforov & Baloch 2019), these are yet to be widely used in clinical practice.

In addition to ultrasonography and fine-needle aspiration biopsy, thyroid function tests including serum thyroid-stimulating hormone (TSH) level are recommended in the investigation of a thyroid nodule (Perros *et al.* 2014, Haugen *et al.* 2016). The role of serum TSH testing is primarily to identify hyperthyroidism caused by a toxic nodule; however, several authors have reported an association between raised serum TSH and thyroid cancer (Boelaert *et al.* 2006, Fighera *et al.* 2015, Zafón *et al.* 2015, Golbert *et al.* 2017) as well as a correlation between serum TSH and aggressiveness of thyroid cancer (Haymart *et al.* 2008, 2009, McLeod *et al.* 2014).

Despite the strong observational basis for an association between serum TSH and thyroid cancer in patients with thyroid nodules, there is significant difficulty in establishing a causal link due to the difficulty in adequately adjusting for confounding factors, such as iodine deficiency, autoimmune thyroid disease and cigarette smoking (Singh *et al.* 1999, Zimmermann & Galetti 2015, Cho *et al.* 2018) and the possibility of reverse causality. This difficulty can be overcome by using genetic epidemiological techniques such as Mendelian randomization (MR), which relies upon the fact that genetic variants predisposing to a certain trait are inherited randomly at conception and are not affected by many confounders acting upon observational associations. The aim of this study was to test the hypothesis that elevated serum TSH has a causal role in the development of benign thyroid nodules and differentiated thyroid cancer, using genetic data from 451,025 participants in the UK Biobank.

## Methods

### Participants

We used data from the UK Biobank, a longitudinal study of 500,000 participants aged between 40 and 69 years who were recruited between 2006 and 2010 (Collins 2012, Sudlow *et al.* 2015). After giving informed written consent, participants gave blood, urine and saliva samples for biomarker measurement and genotyping, as well as having anthropometric measurements at the time of enrolment. In addition, patients filled out demographic and health questionnaires and consented to record linkage with national cancer and death registries as well as the Hospital Episode Statistics (HES) database. UK Biobank has received ethics approval from the National Health Service National Research Ethics Service (ref 11/NW/0382).

Genotyping was performed on DNA extracted from whole blood samples by Affymetrix, using two specially designed SNP arrays with over 95% content overlap. The UKBiobank Axiom array® was used for ~450,000 participants and the UK BiLEVE Axiom array® for 50,000 participants (Welsh *et al*. 2017). Extensive central quality control was carried out by the UK Biobank (Bycroft *et al.* 2018). Genotyping data were subjected to multilevel quality control, with exclusion of sex mismatches (genetic sex different from reported sex), duplicated individuals and outliers of heterozygosity. After these exclusions, as well as those individuals who have subsequently withdrawn from the UK Biobank Study, 451,025 individuals of White European descent were identified using principal components computed from the 1000 Genomes Project. The KING kinship matrix was then used to remove related individuals up to three degrees of separation and identify a subset of 379,708 unrelated individuals for sensitivity analysis. Ancestral principal components were generated among this group of individuals.

### Exposure and outcome measures

We identified two outcome groups of interest within the UK Biobank: those with a diagnosis of differentiated thyroid cancer and those with a diagnosis of benign nodular thyroid disease. In order avoid reporting bias, we discounted self-reported diagnoses in the health questionnaire and used Cancer Registry and HES data only. Thyroid cancer cases were identified by the ICD-10 code ‘C73’. Histology codes were then used to exclude patients with medullary thyroid carcinoma, anaplastic carcinoma, thyroid lymphoma and unclassified subtypes, leaving only patients with differentiated thyroid carcinoma. This resulted in 462 cases. Patients with a diagnosis of benign nodular thyroid disease were identified by the ICD-10 code ‘D34‘. Patients diagnosed with both nodular thyroid disease and thyroid cancer were excluded to avoid bias caused by misdiagnosis (*n* = 147). This left 2031 cases in total. Control groups with no previous diagnosis of cancer and no previous diagnosis of benign thyroid disease were also created, numbering 391,458 and 448,532, respectively.

The exposure of interest in this study was a genetic predisposition to higher TSH levels. In order to quantify this, we utilized 20 SNPs associated with TSH levels at genome wide significance (*P*-value threshold of 5 × 10^−8^) in a meta-analysis of 26,420 individuals of European ancestry across 18 cohorts (Porcu *et al.* 2013) (Table 1). Linkage disequilibrium (LD) was calculated using the LDlink SNPClip application, with an *R*^2^ threshold of 0.1 and a minor allele frequency (MAF) threshold of 0.01 (Machiela & Chanock 2015). No SNPs were removed due to LD. The 20 SNPs have been reported to account for 5.64% of variance in serum TSH levels (Porcu *et al.* 2013). The effect of the included SNPs on thyroid-specific gene expression was investigated using the Genotype-Tissue Expression Consortium tool (www.gtexportal.org) and is shown in Table 1.

**Table 1:** TSH SNPs, their effect sizes on TSH (modified from Porcu *et al*. 2013) and their effect on thyroid-specific gene expression.

Chromosome	Position	Effect/other allele	SNP	Effect size	s.e.	Thyroid-specific gene expression
5	76566105	A/G	rs6885099	−0.141	0.009	No
6	165966473	C/G	rs753760	0.100	0.010	Yes
1	19713761	A/G	rs10799824	−0.113	0.012	Yes
16	78306854	T/C	rs3813582	0.082	0.010	Yes
6	43919740	T/C	rs9472138	−0.079	0.010	Yes
6	44012758	T/C	rs11755845	−0.065	0.010	Yes
4	149888956	T/C	rs10032216	0.087	0.011	Yes
2	217333768	A/G	rs13015993	0.078	0.010	Yes
17	67639131	T/C	rs9915657	−0.064	0.009	Yes
1	61393084	A/G	rs334699	−0.141	0.021	No
15	47533656	A/T	rs10519227	−0.072	0.011	Yes
11	45184143	T/C	rs17723470	−0.065	0.010	Yes
15	86920108	A/G	rs17776563	−0.060	0.010	Yes
19	7174848	T/G	rs4804416	−0.057	0.009	No
9	135129086	A/C	rs657152	0.058	0.009	No
14	92665344	A/C	rs11624776	−0.064	0.011	Yes
8	32535816	A/G	rs7825175	−0.066	0.001	Yes
14	35643769	T/C	rs1537424	−0.052	0.009	Yes
6	148562985	T/C	rs9497965	0.051	0.009	No
9	4257209	A/G	rs1571583	0.057	0.010	No

Positions given are in build 36. Tissue-specific expression information from the Genotype-Tissue Expression Consortium (www.gtexportal.org).

### Data analysis

In order to identify the causal effect of TSH on thyroid cancer and benign nodular thyroid disease, we performed two-sample Mendelian randomization (MR) (Bowden *et al.* 2016*a*) using the 20 known genetic variants associated with TSH (Porcu *et al.* 2013). We corrected for inter-relatedness by performing a GWAS of the thyroid cancer and benign nodular thyroid disease variables using a linear mixed model in the BOLT-LMM software (Loh *et al.* 2015). The 20 known TSH variants were then extracted from these GWAS analyses for use in the two-sample MR. The SNP-TSH association was taken from the primary GWAS by Porcu *et al.*, while the SNP-outcome association was taken from the BOLT-LMM GWAS of our UK Biobank outcome traits. Using the median s.d. (0.8 mIU/L) from the meta-analysis of studies used to identify genetic variants associated with TSH (Porcu *et al.* 2013), the coefficients from the two-sample MR were adjusted to approximate the odds ratios per unit increase in TSH.

MR relies upon the fact that the instrumental variable being used is associated with the risk factor of interest, that the instrumental variable is not subject to the confounding factors acting upon the association between the risk factor and outcome of interest and that the instrumental variable is associated with the outcome of interest *only* via its effect on the risk factor of interest. Figure 1 illustrates the principles of MR.

**Figure 1:** If a risk factor, for example, high TSH truly causes an outcome, for example, thyroid cancer, then the genetic variants for the risk factor should also be associated with the outcome. Unlike the observed risk factor, the genetic variants are not susceptible to confounding by other risk factors or reverse causation (dashed lines) as they are assigned at conception. Horizontal pleiotropy (dotted line), whereby the variants of interest also affect the outcome via their association with another trait is a possible limitation of MR.

Three different methods of two-sample MR were performed. First, inverse variant weighted (IVW) instrumental variable analysis. IVW assumes that all genetic instruments are valid and is therefore susceptible to horizontal pleiotropy (variants affecting the outcome via a route other than the risk factor of interest). To reduce this potential source of bias, we also used the MR-Egger and Median MR techniques (Bowden *et al.* 2016*a*,*b*) which are more robust to pleiotropy. In MR-Egger analysis, the intercept is unconstrained to allow a weighted regression, thus removing the assumption that all variants are valid instrumental variables. This reduces the possibility of variants having a stronger effect on the outcome than the exposure itself (actual TSH levels). Median-MR is also more resistant to pleiotropy, as it uses the median instrumental variable from all included variants and allows for up to 50% of the variants to be invalid.

In order to allow for sensitivity analyses, the effect sizes of the 20 included TSH-associated SNPs were used to produce a genetic risk score (GRS) for TSH in the smaller subset of 379,708 unrelated UK Biobank participants. This group contained 425 cases of differentiated thyroid cancer and 1812 cases of benign nodular thyroid disease. The association between these GRSs and the outcome traits of benign nodular thyroid disease and thyroid cancer was then tested using a logistic regression model with adjustment for age, sex, ancestral principal component and recruitment center. Robust s.e. were used to allow for uncertainty in the estimate. In addition, the 379,708 unrelated participants were divided into quartiles based on their GRS for TSH, and logistic regression analysis was used to test the association between GRS quartile and both disease outcomes. Finally, sensitivity analysis was performed to account for patients with a diagnosis of either hyper- or hypothyroidism as identified in the self-reported health questionnaire or the Hospital Episode Statistics data. A post hoc power calculation using a Mendelian randomization power calculator (Brion *et al.* 2013) confirmed the power of the study to detect a true odds ratio of 4.96 for the binary outcome of benign nodular thyroid disease per 1 s.d. increase in genetically determined TSH (Power = 1.00; α = 0.05; non-centrality parameter = 850.45; F statistic = 26959.26); and a true odds ratio of 2.00 for the binary outcome of thyroid cancer per 1 s.d. increase in genetically determined TSH (Power 1.00; α = 0.05; non-centrality parameter = 113.44; F statistic 26959.26).

## Results

Table 2 displays basic information on the unrelated subgroup of participants and controls. Participants with a diagnosis of benign nodular thyroid disease were more likely than controls to be female, have a higher BMI and have co-existent type two diabetes mellitus (T2DM), hyper- or hypothyroidism. Those with a diagnosis of thyroid cancer were also more likely than controls to be female, and marginally more likely to be obese, with a higher proportion than controls having co-existent hyper- or hypothyroidism.

**Table 2:** Summary of demographic characteristics of participants.

Characteristics	Benign nodular thyroid disease	Controls	*P*-value	Thyroid cancer	Cancer-free controls	*P*-value
*n*	1812	377,896		425	310,176	
Female sex	1492 (82.34)	203,244 (53.78)	<1 × 10^−15^	316 (74.35)	165,537 (53.37)	5.6 × 10^−17^
Mean age at recruitment (s.d.), years	58.92 (7.39)	57.23 (8.01)	<1 × 10^−15^	57.72 (7.29)	56.54 (8.04)	0.0022
Smoking status:						
Never	976 (53.86)	203,242 (53.78)	0.04	233 (54.82)	169,785 (54.74)	0.40
Former	649 (35.82)	133,744 (35.40)		152 (35.76)	107,027 (34.51)	
Current	166 (9.16)	35,774 (9.47)		32 (7.53)	29,261 (9.43)	
Missing	21 (1.16)	5136 (1.36)		8 (1.88)	4103 (1.32)	
Mean townsend deprivation index (s.d.)	−1.16 (3.09)	−1.48 (2.99)	4.8 × 10^−8^	−1.63 (2.94)	−1.45 (2.99)	0.42
Mean units of alcohol (s.d.)	0.20 (1.07)	0.57 (1.04)	2.5 × 10^−6^	0.37 (1.00)	0.57 (1.04)	0.48
Mean BMI (s.d.), kg/m^2^	27.96 (5.23)	27.38 (4.78)	4.1 × 10^−12^	27.55 (5.34)	27.38 (4.77)	0.16
Obese: BMI 30–40 kg/m^2^	471 (25.99)	83,503 (22.10)	1.6 × 10^−9^	111 (26.12)	68,563 (22.10)	0.068
Type 2 diabetes	70 (3.86)	11,996 (3.17)	0.0037	16 (3.76)	9290 (3.0)	0.16
Hypothyroidism	182 (10.04)	18,600 (4.92)	4.8 × 10^−9^	28 (6.59)	15,238 (4.91)	0.12
Hyperthyroidism	59 (3.26)	2897 (0.77)	1.6 × 10^−4^	7 (1.65)	2377 (0.77)	0.35

Table represents data after exclusion of related individuals due to the difficulty in adjusting observational analyses for relatedness. Values stated are numbers (percentages), unless otherwise stated. *P*-values calculated using logistic regression adjusted for age and sex.

### Two-sample MR

Two-sample MR provided evidence that higher TSH caused both benign nodular thyroid disease and thyroid cancer. A 1 s.d. (approximately 0.8 mIU/L) higher genetically instrumented TSH level was associated with 4.96 higher odds of benign nodular thyroid (95% CI 2.46–9.99) and 2.00 higher odds of thyroid cancer (95% CI 1.09–3.70; Fig. 2 and Table 2). This approximates to 7.39 times higher odds of benign nodular thyroid disease (95% CI 3.67–14.90) and 2.39 times higher odds of thyroid cancer (95% CI 1.29–4.40) per 1 mIU/L higher TSH. The more pleiotropy-resistant two-sample analyses were directionally consistent and MR-Egger provided no evidence of horizontal pleiotropy for either outcome trait (Table 3).

**Figure 2:** Forest plot showing two sample MR (instrumental variable analysis) associations between genetically instrumented TSH and thyroid cancer and benign nodular thyroid disease. Odds ratios of outcome per s.d. higher genetically instrumented TSH and 95% CIs are shown.

**Table 3:** Results of two-sample MR analysis for benign nodular thyroid disease and thyroid cancer.

Trait	IVW		Egger			WM		PWM	
	OR (95% CI)	*P*-value	OR (95% CI)	*P*-value	Int *P*	OR (95% CI)	*P*-value	OR (95% CI)	*P*-value
Thyroid cancer	2.00 (1.09–3.70)	0.039	1.71 (0.23–12.72)	0.60	0.87	1.88 (1.04–3.39)	0.037	1.50 (0.83–2.73)	0.18
Benign nodular thyroid disease	4.96 (2.46–9.99)	2.59 × 10^−4^	1.46 (0.16–13.43)	0.74	0.27	3.84 (2.27–6.49)	5.54 × 10^−7^	5.44 (2.90–10.21)	1.37 × 10^−7^

Beta coefficients and *P* values for the inverse variant weighted (IVW), Egger, weighted median (WM) and penalised weighted median (PWM) analyses are displayed. Int *P* represents the *P*-intercept of Egger analysis, which is a measure of horizontal pleiotropy. s.e. are displayed in parentheses.

### Sensitivity analyses

The GRS for TSH was associated with both benign nodular thyroid disease and thyroid cancer in the subgroup of unrelated participants. Using logistic regression adjusted for age, sex, ancestral principal component and assessment center with the GRS for TSH as the dependent variable, we found a positive association with benign nodular thyroid disease, with each weighted allele increase in the TSH GRS resulting in 1.11-fold higher odds of benign nodular thyroid disease (95% CI 1.10–1.13; Fig. 3). Similarly, there was a positive association with thyroid cancer, with an odds ratio of 1.05 (95% CI 1.02–1.09; Fig. 3). Furthermore, individuals in the top 25% of the TSH GRS were at 1.34 higher odds of thyroid cancer (95% CI 1.14–1.50; Fig. 4) and 2.23 higher odds of benign nodular thyroid disease (95% CI 1.89–2.63) than those in the bottom 25%. Results of the sensitivity analysis after excluding participants with hypothyroidism or hyperthyroidism, which did not affect the associations, are shown in Table 4. Finally, the analysis using TSH GRS in the unrelated subgroup was repeated separately in male and female participants (Table 5) with the associations with both benign nodular disease and thyroid cancer remaining stable in females, but the association with thyroid cancer weakening in males.

**Figure 3:** Forest plot showing associations between genetically instrumented TSH and thyroid cancer and benign nodular thyroid disease. Odds ratios of outcome per s.d. higher genetically instrumented TSH and 95% CIs are shown.

**Figure 4:** Forest plot showing associations between quartiles for TSH genetic risk and thyroid cancer and benign nodular thyroid disease. Odds ratios and 95% CIs are shown for each quartile as compared to those in the lowest quartile.

**Table 4:** Results of sensitivity analysis for both thyroid cancer and benign nodular thyroid disease after exclusion of participants with co-existing diagnoses of hypothyroidism or hyperthyroidism.

Analysis	Exposure	OR thyroid cancer	*n* = cases (controls)	95% CI	OR Benign nodular thyroid disease	*n* = cases (controls)	95% CI
Primary analysis	TSH	1.05	425 (310,176)	1.02–1.09	1.11	1812 (377,896)	1.10–1.13
Sensitivity analysis	TSH	1.05	423 (309,526)	1.02–1.09	1.13	1803 (377,110)	1.11–1.14

**Table 5:** Results of sensitivity analysis for both thyroid cancer and benign nodular thyroid disease according to sex.

Analysis	Exposure	OR thyroid cancer	*n* = cases (controls)	95% CI	OR Benign nodular thyroid disease	*n* = cases (controls)	95% CI
Primary analysis	TSH	1.05	462 (391,458)	1.02–1.09	1.11	1812 (377,896)	1.10–1.13
Male sex	TSH	1.01	109 (144,639)	0.94–1.08	1.12	320 (174,652)	1.08–1.15
Female sex	TSH	1.07	316 (165,537)	1.03–1.11	1.13	1492 (203,244)	1.11–1.15

## Discussion

### Principal findings

This study investigated the causal relationship between serum TSH levels and thyroid cancer risk and benign nodular thyroid disease risk. Our results reveal a significant association between genetic variants predicting higher serum TSH and both diagnoses. Furthermore, these results were consistent when using different approaches.

The first study to identify an association between serum TSH levels and risk of thyroid cancer was published by Boelaert *et al.* (2006) and since then many authors have reported similar findings, with two meta-analyses reporting positive associations (McLeod *et al.* 2012, Zheng *et al.* 2016). However, the majority of included studies were retrospective, resulting in bias and difficulty in adjusting for all confounders. There is also some controversy on the subject, with the EPIC case-control study reporting a negative association among its 357 cases and 767 matched controls (Rinaldi *et al.* 2014), and a more recent case-control study on papillary thyroid carcinoma identifying a positive association in men and a negative association in women (Huang *et al.* 2017). Furthermore, differentiated thyroid cancer has been reported even in patients with completely suppressed TSH levels (Satta *et al.* 1993), although the authors note that tumors may have arisen prior to development of thyrotoxicosis. Here, we demonstrated stronger evidence of a role for TSH in thyroid cancer in women than in men. However, these analyses were limited by the low numbers of male participants with thyroid cancer in the UK Biobank study. When testing the role of TSH on benign thyroid nodules, results were similar in men and women.

The widely proposed mechanism explaining the positive association between serum TSH levels and both benign thyroid nodules and thyroid cancer reported by most studies is the thyrotropic effect of TSH. TSH is known to induce proliferation of thyrocytes and both benign and malignant thyroid tumors have long been known to express TSH receptors (Ichikawa *et al.* 1976). Furthermore, suppression of TSH is a well-established adjunct to the management of differentiated thyroid carcinoma (Perros *et al.* 2014) and has in the past been used in the treatment of benign nodular thyroid disease although has now largely been abandoned in this setting due to long-term adverse effects (Wémeau *et al.* 2002). Animal studies have demonstrated a convincing role for TSH in thyroid tumorigenesis (Lu *et al.* 2010) however the cause-effect relationship between high TSH and thyroid cancer in humans is unclear due to the difficulty in accounting for known and unknown confounders.

The aim of this study was to test the hypothesis that TSH has a causal role in the development of thyroid cancer, using genetic techniques. Our findings while positive, are not sufficient to change clinical practice. They do, however, add to the debate on the topic and represent evidence using a novel technique that higher TSH does increase the risk of both benign nodular thyroid disease and thyroid cancer. It is vital that this causal relationship is understood when considering previously published observational and clinical studies on the link between TSH and thyroid cancer. Furthermore, our findings help pave the way for future research on the ability of genetic instruments to distinguish between benign and malignant thyroid nodules, with the advantage that they are not confounded by environmental factors. This information may eventually be used along with other genetic instruments to formulate pre-diagnostic screening or stratification tools to aid clinical decision making in patients with thyroid nodules.

### Strengths and limitations

The advantage of the present study is the ability to limit the effect of environmental confounders by using genetic predictors of TSH levels, which are fixed at conception. This is the first study using Mendelian randomization to investigate the link between TSH levels and benign nodular thyroid disease and thyroid cancer. The main limitation of the study is the lack of an observational measure of TSH in the UK Biobank cohort. This problem is partially overcome by using data from large genome wide association studies to confirm robust associations between the TSH SNPs we used and TSH levels in European subjects; however, the UK Biobank participants are inevitably not completely comparable to those cohorts. Secondly, the power of our MR analyses is somewhat limited by the small number (462) of thyroid cancers amongst the UK Biobank participants. Finally, the UK Biobank is not representative of the wider population, including only UK residents aged between 40 and 69 at enrolment. There is some evidence of healthy volunteer bias within the UK Biobank, with lower rates of cancer incidence than the age and sex matched general population (Fry *et al*. 2017).

### Conclusions

Using MR, we have demonstrated a causal role for TSH in both benign nodular thyroid disease and differentiated thyroid cancer. This supports the associations reported by many observational studies. Further research is required to test the applicability of these findings to the wider population and investigate their clinical applicability in patients with thyroid nodules.

## Declaration of interest

The authors declare that there is no conflict of interest that could be perceived as prejudicing the impartiality of the research reported.

## Funding

J T is supported by an Academy of Medical Scienceshttp://dx.doi.org/10.13039/501100000691 (AMS) Springboard award, which is supported by the AMS, the Wellcome Trusthttp://dx.doi.org/10.13039/100010269, GCRF, the Government Department of Business, Energy and Industrial strategy, the British Heart Foundationhttp://dx.doi.org/10.13039/501100000274 and Diabetes UK (SBF004/1079). R N B is supported by a Wellcome Trusthttp://dx.doi.org/10.13039/100010269 and Royal Society grant (WT104150).
